This article has been retracted.

# The Healing Effects of Piano Practice-Induced Hand Muscle Injury

**DOI:** 10.1155/2022/1020504

**Published:** 2022-07-18

**Authors:** Hecheng Yu, Xiaoming Luo

**Affiliations:** ^1^Department of Rehabilitation Medicine, Affiliated Tenth People's Hospital of Tongji University, Shanghai Tenth People's Hospital, China; ^2^Department of Physical Therapy, Affiliated Yangzhi Rehabilitation Hospital of Tongji University, Shanghai Yangzhi Rehabilitation Hospital, China

## Abstract

**Background:**

The muscles related to piano practice are mainly concentrated in the fingers and upper limbs, and the muscles related to other parts of the body are weak. Compared with other sports injuries, the injuries caused by piano practice are mainly chronic injuries caused by long-term strain of the upper limbs, and acute injuries rarely occur. The purpose of this study was to analyze the therapeutic effect of hand muscle injury caused by piano practice.

**Method:**

A total of 60 patients with hand muscle injury caused by piano practice admitted to our hospital from January 2019 to June 2020 were selected. According to the number random grouping method, they were randomly divided into two groups. There were 30 patients in the observation group, including 20 males and 10 females, aged 24-53 (39.51 ± 7.01) years old, and the course of disease was 1-5 (3.24 ± 1.62) months. In the control group, there were 30 patients, including 18 males and 12 females, aged 24-56 (39.62 ± 7.17) years old, and the course of disease was 1.5-5 (3.14 ± 1.71) months. If the observation group experienced excessive pain, the group took ibuprofen sustained-release capsules. On weekdays, exercise your fingers 2-3 times per day. After the intervention, the wrist joint function score of the observation group was higher than that before the intervention.

**Results:**

Before treatment, there was no significant difference in pain level scores between the two groups (*P* > 0.05). After treatment, the limb pain score in the observation group was lower than that in the control group. The effective rate of hand tendon rehabilitation in the observation group was 93.33%. The effective rate of hand tendon rehabilitation in the control group was 70.00%. The comparison results showed that there was statistical significance (*P* < 0.05). The score of the observation group was significantly higher than that of the control group, with statistically significant differences (*P* < 0.05).

**Conclusion:**

Piano workouts can cause hand muscle difficulties, which can be alleviated by daily finger gymnastics. Daily finger exercises are simple and not limited by time and place. Piano practitioners can use the spare time of daily training and performance to exercise for a long time, so as to prevent or recover finger muscle damage caused by piano practice. It has the potential to help pianists avoid hand muscle injuries when practicing while also allowing music to reach its full potential.

## 1. Introduction

The upper limb muscles help us move our arms and hands under the command of our brain. Muscles can only exert force in one direction since they contract. Two muscles or two sets of muscles are required to move a bodily part in two directions, one to move it one way and the other to move it the other. Therefore, the movement of muscle has the characteristics of unidirectional [1, 2]. Piano practice involves ten fingers, arms, shoulders, and neck muscles. It is an upper limb movement coordinated by many muscle groups [3]. To allow movement, the opposing muscle must relax and extend in response to the contraction of one muscle. If this does not occur, that is, if the opposing muscle stays tense—both muscles contract at the same time, which is known as cocontraction. Cocontraction is a movement-inhibiting condition that can result in damage [4, 5]. Piano practice is a long-term, fast-paced upper limb movement. During piano practice, the upper limb muscles are in a high load contraction state for a long time [6]. Tense exercise causes muscle contraction for a long time, coupled with the irregularity of piano practice, which is the main source of muscle injury [7]. There are many factors that affect human muscle health: reasonable rest, adequate sleep, age growth, and scientific exercise and prevention [8]. This explains why some pianists can perform for years without incident before suffering an injury in their late thirties or forties. They are not playing any differently, but their bodies are less able to handle the stress. The finger flexor system, which is located in the top half of our lower arm around the elbow, controls the majority of finger movements [9, 10]. The interosseous muscle system is the second muscular system that regulates finger mobility. The interphalangeal muscles and the interosseous dorsal muscles are interosseous muscles that are dispersed across the palm [11]. Modern piano playing necessitates playing with the upper arm's gravity pull, with a focus on simple, sharp movements of the small muscles of the fingers and synchronised, relaxed motions of the upper body, shoulders, and arms [12, 13]. The muscle energy of the human body structure must be used to develop piano skills. It is simple to make training blunders and permanently injure human body muscles without this foundation [14]. The following are the results of 60 cases of hand muscle injury induced by piano practice that were collected and treated in this research. The specific chapter structure is shown in Figure 1.

## 2. Materials and Methods

### 2.1. General Information

A total of 60 patients with hand muscle injury caused by piano practice from January 2019 to June 2020 were selected and considered two research groups. The observation group included 20 males and 10 females, aged 24-53 (39.51 ± 7.01) years old, and the course of disease was 1-5 (3.24 ± 1.62) months. The control group included 18 males and 12 females, aged 24-56 (39.62 ± 7.17) years old, and the course of disease was 1.5-5 (3.14 ± 1.71) months. Details of the two groups are shown in Table 1.

In this study, we took the wrist and fingers as the whole research part. Because the muscle injury caused by piano practice has certain particularity, the inclusion criteria and exclusion criteria are formulated on the premise of diagnostic criteria.

1. Diagnostic criteria: according to the conscious symptoms of the wrist (positive for any of the acid, numbness, or tingling of the finger or wrist) and check the signs of the hand (positive for swelling or atrophy of the musculus magnus) [15], and the diagnosis was confirmed according to the relevant diagnostic criteria of practical neurological diseases and therapeutics [16]
2. Inclusion criteria: ① meeting the diagnostic criteria of hand muscle injury caused by piano practice; ② voluntary subjects signed informed consent; ③ oral medication or external application of traditional Chinese medicine in strict accordance with the doctor's advice; ④ cooperating with the collection of test results, compliance was good
3. Exclusion criteria: ① those who had taken oral analgesics or local physiotherapy before treatment to affect the efficacy evaluation; ② local skin rupture; ③ suffering from cervical spondylosis or other diseases that cause shoulder pain, such as intrashoulder joint fractures, tuberculosis, bone metastases, and other diseases that affected shoulder joint mobility; ④ acute phase with severe liver and kidney dysfunction, heart disease, endocrine disease, and other diseases

### 2.2. Methods

#### 2.2.1. Control Group

The treatment method of the control group is to use drugs only to relieve pain; other methods of rehabilitation with fingers and wrists are not assisted. Among them, ibuprofen sustained-release capsules produced by Sino US joint venture Tianjin Shike Pharmaceutical Co., Ltd. were selected as the analgesic drugs: production batch number: National Pharmaceutical Standard H20013062, specification 0.4 g, 1 capsule per time, taking it orally once in the morning and evening after meals, taking it with warm water after meals, and continuing treatment for 15 days. During this process, record the time from taking the medicine to pain relief, the degree of pain and the duration of pain, and the number of intermittent pain every day (including acid swelling and other finger and wrist discomfort).

#### 2.2.2. Observation Group

In the observation group, the pain of the participants was first evaluated. If the pain was tolerable, they would not take drugs, and only use the finger exercise method proposed in this study. If the pain is too great, you can take ibuprofen sustained-release capsules to relieve the pain and continue to exercise your fingers 2-3 times a day for six months. Finger exercises include ① arm relaxation exercises, ② finger push-ups, and ③ wrist spring operation. Specific exercises related to the hands are shown in Figure 2.

1. Arm relaxation exercises: stand naturally with shoulders relaxed and falling. Then, bend elbows slightly and raise arms naturally to shoulder height. Hold for 2 or 3 seconds and let the whole arm fall into free fall. After practicing several times, alternate left and right hands to drop and lift. Then, make further adjustments to this exercise: slowly raising hands to head height. Hold for 2 or 3 seconds and then lower arms slowly and controllably. When reaching shoulder height, immediately relax and fall [17]. It should be noted that the relaxation should be carried out in an instant as much as possible and should not be gradually adjusted to a relaxed state. Let the slight tension control and the complete relaxation exercise combine to improve the ability of arm tightness adjustment
2. Finger push-ups: the training steps were as follows: stand upright, facing the wall, about two-thirds of the arm away from the wall; stand each finger separately on the wall, the palm joints protruding, the palms arched, the wrists slightly lower than the palm joints [18]. Then, slowly lean forward, bending elbows and letting weight pour into fingertips and toes to increase their support. After the weight pressure reached the appropriate level, stay for 2 or 3 seconds, slowly push away until the body was upright and return to its original state; let arms down and relaxed a little. Repeat this exercise
3. Wrist spring operation: sit with body upright, shoulders and arms relaxed, elbows bent to about 90 degrees to play close to the body; relax the wrist and open the fingers naturally so that there was about an octave distance between the fingers, 2, 3, 4 fingers slightly raised in an arched hand shape. Then, keep the wrists and elbows of both hands at the original height, with the palm part facing the body direction, which was the upper part of the oblique after instant force, for a quick spring [19]. After that, relax completely and let hands fall naturally. This movement was just like the daily action of knocking on the door with the finger joints. Its force was mainly to bounce upwards. The three joints were used as the central fulcrum of the force to bounce, and the force was quickly concentrated and then relaxed instantly

### 2.3. Selection of Indicators

After 6 months of treatment, the pain degree, joint mobility, and daily activities of the two groups were compared.

1. The degree of pain: using NRS [20] (NRS is a scoring system for pain; the score range is 0-10 points, of which 0-3 points belong to mild pain, 4-7 points belong to moderate pain, and 8-10 points belong to severe pain) to assess the patient's shoulder pain, the scale used 0 to 10 points to represent different degrees of pain; 0 pointed to no pain, 10 pointed to unbearable severe pain, and the middle part indicated different degrees of pain, and it was evaluated once before and after treatment
2. Joint mobility: standard for measuring total active range of motion (TAM is a scoring system for evaluating the overall function of the palm advocated by the final results Committee of the American Society of Hand Surgery; TAM is the sum of the angles formed by the maximum flexion of the metacarpophalangeal joint, proximal and distal interphalangeal joints in the fist grip position minus the sum of the limited extension of these joints) [21]: excellent rehabilitation: TAM > 220; good recovery: TAM200~220; poor rehabilitation effect: TAM < 180
3. Ability to perform daily activities: both groups were assessed with the Daily Living Activity Scale (FIM, the main evaluation index of FIM is self-care activities, including the impact of walking and hand movement on life) [22]; there were 7 points for each item, a total of 42 points

### 2.4. Statistical Methods

Using SPSS 19.0 statistical software for data analysis, measurement data in line with the normal distribution were expressed as *X* ± *S*. The comparison between groups was performed by *t*-test, statistical data were compared by using the *χ*^2^ test, and *P* < 0.05 meant the difference was statistically significant.

## 3. Results

This section follows the relevant standards proposed in the previous section, collates the two groups of data based on the three indicators: pain level, joint range of motion, and daily activity ability, and compares the results.

### 3.1. Results of Pain Level

There was no significant difference in pain level scores between the two groups (*P* > 0.05) before treatment. The limb pain score in the observation group was lower than that of the control group after treatment. Results of pain level are shown in Table 2.

### 3.2. Results of Joint Range of Motion

The effective rate of hand tendon rehabilitation in the observation group was 93.33%. The effective rate of hand tendon rehabilitation in the control group was 70.00%, and the comparison results showed that there was statistical significance (*P* < 0.05). Results of joint range of motion are shown in Table 3.

### 3.3. Results of Daily Activity Ability

There was no difference in daily living ability scores between the two groups (*P* > 0.05), after treatment and before treatment. The scores of washing, wearing a jacket, going to the toilet, eating, bathing, and wearing pants in both groups were all improved. Results of daily activity ability are shown in Table 4.

## 4. Discussion

Piano playing is a highly repetitive activity. The players sit for a long time, their upper limb muscles tense and contract during training and performance, and their wrists and fingers move fast, which brings great hidden dangers to the hand muscle injury of piano players [23]. Some scholars have done experiments to set the metronome at a quarter-note equal to 120 tempo, and the number of repetitions for playing a sixteenth-note one hour continuously is 28,800 times. It is only an hour, and with a little more effort, eight hours a day for more than twenty years, it can imagine how many times our fingers would repeat the work [24, 25]. Piano playing is another highly technical activity. It must be improved after thousands of times of practice. “Repetition” is unavoidable for every piano learner [26]. Highly repetitive performance is a prerequisite for the formation of performance sports injury. Piano skills training must be based on the body structure and muscle energy. Different trainees have their own characteristics in the hand muscle energy structure. They cannot be the same. Training should maximize strengths and avoid weaknesses. At the same time, when practicing the piano, the trainer should consider his own physical condition and avoid excessive exercise for a long time [27]. Modern piano playing requires the player to use hand muscles to coordinate the relaxed upper body and shoulder and arm muscles. How to find a way to relax the muscles while practicing and playing is a challenge that every piano practitioner needs to face [28]. In order to achieve natural, relaxed, and touching performance, players need to adopt macro comprehensive adjustment and micro detail control [29]. Macro comprehensive regulation requires piano players to pay attention to the prevention of hand muscle injury and pay attention to scientific rehabilitation methods after hand muscle injury. We should not blindly rely on drugs for pain relief. Drug pain relief has the characteristics of short term and temporary, so we cannot achieve the basic rehabilitation goals, nor can we keep a fluke mentality [30]. In the absence of external intervention, it is difficult to self-heal the hand muscle injury caused by piano training [31]. If it is not handled properly, it will not only affect the pianist's performance level but also have a great chance to leave sequelae such as finger joint deformation, tenosynovitis, and cervical spondylosis [32, 33]. Micro comprehensive adjustment requires piano players to formulate scientific and reasonable practice time and methods when preventing hand muscle injury. After hand muscle injury, go to the hospital for examination in time. With the help of doctors, formulate scientific health care plans and methods and reserve sufficient hand rest time. Pay attention to relaxing muscles while playing and training, and do scientific hand exercises between playing and training [34].

There was no significant difference in pain level scores between the two groups (*P* > 0.05) before treatment, and the limb pain score in the observation group was lower than that of the control group after treatment. The effective rate of hand tendon rehabilitation in the observation group was 93.33%. The effective rate of hand tendon rehabilitation in the control group was 70.00%; the comparison results showed that there was statistical significance (*P* < 0.05). Before treatment, there was no significant difference in daily living ability scores between the two groups (*P* > 0.05). After treatment, the scores of washing, wearing a jacket, going to the toilet, eating, bathing, and wearing pants in both groups were all improved. However, the observation group's limb pain score was lower than the control group's, and the observation group's wrist hand function score was higher than the control group's.

## 5. Conclusion

Through the above research, we draw the following three conclusions:

1. Hand muscle injury is a common sports injury for piano players, which has the characteristics of high incidence and inevitability. The rehabilitation period of injury is long, which has a great impact on the life of piano practitioners
2. ① Arm relaxation exercises, ② finger push-ups, and ③ wrist spring operation: three kinds of body movements are of great help to the rehabilitation of piano players' muscle injuries
3. Daily finger exercises are simple and not limited by time and place. Piano practitioners can use the spare time of daily training and performance to exercise for a long time, so as to prevent or recover finger muscle damage caused by piano practice

## Figures and Tables

**Figure 1:** Structure of this study.

**Figure 2:** Main contents of finger motor rehabilitation.

**Table 1:** General information.

Groups	Cases	Gender		Age	Course of disease (month)
		Males	Females		
Observation group	30	20	10	39.51 ± 7.01	3.24 ± 1.62
Control group	30	18	12	39.62 ± 7.17	3.14 ± 1.71

**Table 2:** Results of pain level.

Groups	Cases	Limb pain VAS		Wrist hand function VAS	
		Before	After	Before	After
Observation group	30	4.15 ± 1.28	2.01 ± 1.09	51.02 ± 17.61	73.06 ± 15.74
Control group	30	4.20 ± 1.34	3.52 ± 1.31	50.36 ± 16.22	70.05 ± 14.91

**Table 3:** Results of joint range of motion.

Groups	Cases	Excellent TAM	Good TAM	Poor TAM	Rate
Observation group	30	16	12	2	93.33
Control group	30	9	12	9	70.00

**Table 4:** Results of daily activity ability.

Groups	Time	Washing	Wearing a jacket	Going to the toilet	Eating	Bathing	Wearing pants	Total
Observation group	Before	3.18 ± 1.07	3.27 ± 1.09	3.17 ± 1.02	3.06 ± 1.04	3.09 ± 1.35	3.09 ± 1.48	19.08 ± 3.57
	After	6.38 ± 0.36	6.07 ± 0.65	6.23 ± 0.52	6.32 ± 0.63	6.78 ± 0.114	6.38 ± 0.23	35.23 ± 7.01
Control group	Before	3.01 ± 1.11	3.15 ± 1.21	3.23 ± 1.52	3.22 ± 1.01	3.26 ± 1.61	3.04 ± 1.71	18.23 ± 4.62
	After	5.64 ± 0.52	5.34 ± 0.33	5.60 ± 1.20	5.41 ± 1.256	5.33 ± 1.01	4.76 ± 1.01	30.45 ± 8.03

## Data Availability

The data used to support the findings of this study are included within the article.
